RETRACTED

# Cloud Computing to Tourism Economic Data Scheduling Algorithm under the Background of Image and Video

**DOI:** 10.1155/2022/3948221

**Published:** 2022-07-21

**Authors:** Heqing Zhang, Yilin Feng, Leilei Wang

**Affiliations:** ^1^Management (Tourism) School of Guangzhou University, Guangzhou 510006, Guangdong, China; ^2^Universiti Teknologi Malaysia, Skudai 81310, Johor Bahru, Johor, Malaysia

## Abstract

With the rapid development of image video and tourism economy, tourism economic data are gradually becoming big data. Therefore, how to schedule between data has become a hot topic. This paper first summarizes the research results on image video, cloud computing, tourism economy, and data scheduling algorithms. Secondly, the origin, structure, development, and service types of cloud computing are expounded in detail. And in order to solve the problem of tourism economic data scheduling, this paper regards the completion time and cross-node transmission delay as the constraints of tourism economic data scheduling. The constraint model of data scheduling is established, the fitness function is improved on the basis of an artificial immune algorithm combined with the constraint model, and the directional recombination of excellent antibodies is carried out by using the advantages of gene recombination so as to obtain the optimal solution to the problem more appropriately. When the resource node scale is 100, the response time of EDSA is 107.92 seconds.

## 1. Introduction

With the popularization of cloud computing and mobile Internet, more and more business and data storage are carried out in the cloud. Cloud computing applications are constantly infiltrating and developing in all walks of life. Based on cloud computing technology, individual users and small- and medium-sized enterprises can obtain computing, storage, network, and platform services at low cost through Internet services to solve their own problems such as limited funds. They obtain the service resources required by individuals or enterprises with low-cost resource investment, save the cost of building data centers and infrastructure, and reduce the cost of building and maintaining data centers. In this business service model, users should not only consider processing time and efficiency when choosing a service but also consider the economic cost involved in using the service. The economic costs associated with services are mainly determined by factors such as resource consumption and market supply and demand for the provision of corresponding services. Under normal circumstances, cost-sensitive individual users and enterprises will consider economic factors and give priority to lower-cost service resources to complete the corresponding data. For users with higher service quality requirements, they strive to complete data in the shortest time and will choose service resources with strong data processing capabilities. When scheduling in the cloud environment, it is necessary to take into account the economic cost and the quality of service provided to meet the needs of users to the greatest extent.

RETRACTED

Due to the diversification and resource-sharing nature of cloud computing systems, and their large user group, the amount of data that needs to be processed at the same time in the cloud environment is extremely large. Therefore, reasonable and efficient scheduling of resources and data in the cloud environment, ensuring user service quality, and improving user data execution efficiency and resource utilization efficiency are the focus and difficulty in cloud computing technology research. In a cloud computing system, physical resource nodes are heterogeneous. The state of the node will change dynamically with the invocation of the resource. In addition, data scheduling in different application scenarios has different characteristics, resulting in extremely high complexity of scheduling algorithms in the cloud environment. Therefore, for specific application scenarios, an effective data scheduling strategy is formulated according to the characteristics of the corresponding scenarios. Establishing a reasonable mapping between data nodes and resource nodes can shorten data execution time and improve data execution efficiency.

The innovation of this paper is as follows:

1. It introduces the current research status of data scheduling in cloud environment. On the basis of the existing research results, it analyzes specific application scenarios, proposes a reasonable solution according to the influencing factors of the corresponding scenario, and expounds on the theoretical knowledge used in the solution.
2. Aiming at the influence of the regional distribution of resources on the communication transmission between data nodes in the process of tourism economic data scheduling, this paper considers the impact of completion time and cross-node transmission delay on the scheduling strategy in the process of tourism economic data scheduling. It establishes an optimization model of tourism economic data scheduling and utilizes the advantages of artificial immune algorithm in cloud environment data scheduling. The fitness function of the improved artificial immune algorithm is generated by the constraints of the optimization model of tourism economic data scheduling, and the antibodies with lower fitness are directionally mutated in the antibody mutation stage of the algorithm. It is transformed into a better antibody by genetic manipulation to generate the optimal solution to the problem.

RETRACTED

## 2. Related Work

Many scholars have provided a lot of references for research on image video, cloud computing, tourism economy, and data scheduling algorithms.

Chen proposed two dynamic scheduling algorithms for the fog computing scheme of in-vehicle network data scheduling. These algorithms can dynamically adapt to changing network environments and improve efficiency. For performance analysis, a combined formal approach called performance evaluation process algebra is applied to model scheduling algorithms in fog-based vehicle networks [1].

Verma has proposed an adaptive block scheduling (A-CMT) for CMT. Simulation results show that the method achieves better performance in throughput. File transfer times and congestion windows grow. The proposed method improves the average throughput by 13% [2].

Dang proposed a novel real-time data scheduling method based on deep learning and an improved fuzzy algorithm for flexible operation in paper workshops. The algorithm is divided into three parts. The first part describes the flexible job-shop scheduling problem. The second part builds the fuzzy scheduling model of flexible job data in the paper workshop. Finally, the third part uses the genetic algorithm to obtain the optimal solution for the fuzzy scheduling of flexible job data in the papermaking workshop [3].

Luo proposed a unified accurate algorithm based on dynamic programming. This exact algorithm is then developed into a complete polynomial-time approximation scheme for the complementary problem and a dual complete polynomial-time approximation scheme for the original problem [4].

Joo studied the joint scheduling problem of multichannel data transmission and wireless power transmission. The joint problem is formulated using a unified framework, and new difficulties for efficient resource allocation are identified [5].

Zhang studied the problem of efficient flow scheduling in data centers, focusing on elephant flows. By applying stable matching theory, the scheduling problem is modeled and proven to be NP-Hard [6].

Huang proposed a hybrid scheduling model. Combining priority queues with packet general-purpose processor sharing provides diverse quality of service guarantees for multimedia applications in software-defined networks. Network calculus is applied to develop modeling and analysis techniques to evaluate the proposed quality of service performance scenarios. Huang J identified the performance bounds guaranteed by the proposed heterogeneous data flow scheme, including its worst-case end-to-end latency and queuing backlog [7].

RETRACTED

Durazo-Cardenas I developed a proof-of-concept demonstrator to validate system principles and test algorithm functionality. It employs dashboards to visualize system responses and present key information. Real orbital events and inspection datasets are analyzed to issue degradation alerts and initiate automatic scheduling of maintenance tasks [8].

The data from these studies are not comprehensive, and the results of the studies are open to question. Therefore, it cannot be recognized by the public and thus cannot be popularized and applied.

## 3. Cloud Computing

With the advancement of informatization and digitization, the amount of information involved in various fields is gradually accumulating and expanding. Traditional IT facilities have been unable to meet people's demand for information processing performance and speed. Virtualization technology has gradually matured, and network broadband has been continuously developed and accelerated. Internet applications are rapidly expanding in various fields. And the development of big data technology requires a lot of resource performance. In such a social environment, cloud computing technology emerges and develops rapidly in applications [9, 10].

Cloud computing is a type of distributed computing, which refers to decomposing huge data computing and processing programs into countless small programs through the network “cloud.” Then, these small programs are processed and analyzed through a system composed of multiple servers, and the results are obtained and returned to the user. In the development process of cloud computing, because different enterprises have different understandings of cloud, the business and service objects are also different. Therefore, the adopted cloud computing solution architecture will be different, and there is no unified standard for the corresponding architecture [11, 12]. A comparative study is made on the cloud computing solution architectures of different enterprises. Although these architectures are different in form, they are essentially the same, only the difference in form. In general, the architecture of cloud computing can be represented as shown in Figure 1 [13, 14]. Cloud computing is characterized by virtualization technology, dynamic scalability, on-demand deployment, high flexibility, and high reliability [15, 16].

1. *Resource Layer*. This layer is mainly based on the types of virtualized resources such as computing, storage, and network provided by physical resources. It is available to cloud users as a service. When users use this layer of services, they only need to provide information such as resource requirements and configuration, and then they can use this layer of resources [17, 18].
2. *Platform Layer*. Users can build applications at this layer, use the middleware services and database services provided by the platform to develop and deploy their own applications, and expand data processing capabilities. Using the services provided by this layer does not need to manage the underlying resources; just upload and deploy personal programs and data using the tools provided by the platform [19, 20].
3. *Application Layer*. This layer mainly provides software services. Enterprises and individuals can rent software services provided by the cloud platform to solve their own information management problems, such as enterprise e-mail services and financial services. Using the software service at the application layer can save the maintenance and management of the software server, which is convenient and efficient [21, 22].
4. *Access Layer*. The cloud platform provides users with a variety of interfaces to access services, such as web portals, web services, and command lines. Users can view the service catalog provided by each layer of the platform according to their own needs and subscribe to management and services on-demand [23, 24].
5. *Monitor Management*. This layer provides management of various services of the platform, management and monitoring of platform security, deployment management of services, and so on to ensure the stability and security of services provided by the platform [25].

RETRACTED

The service types of cloud computing are shown in Figure 2.

1. Infrastructure as a Service (IaaS).
2. IaaS provides cloud users with on-demand physical and virtual resource services, such as servers, storage, and network services. A typical IaaS service is Amazon EC2/S3 [26]. Amazon is the first company to provide cloud computing products. EC2 can provide virtual machine-based resource services. EC2 has product types with different performance and price, and users can choose corresponding services according to their own needs and economic factors. S3 provides simple storage services and can be used for mass information storage.
3. Platform as a Service (PaaS).
4. PaaS can provide a development and deployment environment based on a cloud platform, and users can use this platform to develop their own application software. And users can also provide services to other users with their own application software. In the use of this platform, there is no need to pay attention to the management and maintenance of the underlying resources; just use the services provided by the platform according to the provided specifications. Typical PaaS include Microsoft Windows Azure, and Google APPEngine.
5. Software as a Service (SaaS).
6. The cloud platform provides SaaS services through the network. Enterprises and individuals can use and manage the application software provided by the platform through the network according to their business needs. Typical ones are SalesforceCRM and Google Apps. SalesforceCRM provided by Force.com can provide enterprise management software for enterprise users. It can provide personalized services according to the characteristics of enterprises to formulate corresponding management content. Google Apps provides word processing and mail services. Individuals and businesses can pay to try out the cloud services provided by Google, without worrying about the management and maintenance of the mail service.

RETRACTED

There are four types of cloud platform deployments:

1. *Public Cloud*. Cloud users pay to try the public cloud through the web, which can reduce the operating cost of IT. However, compared with other cloud types, public cloud has shortcomings in terms of security. Data and applications on public clouds are more vulnerable [27].
2. *Private Cloud*. The use of private cloud can make it easier to manage, maintain, and deploy security within the enterprise. Compared with public cloud, it has stronger security.
3. *Hybrid Cloud*. It links one or more external cloud services in the private cloud, which can effectively control the security information used internally and occasionally request the resources of the public cloud [28].
4. *Community Cloud*. One type of cloud that is shared and built by many organizations and user groups is called a community cloud. It can be managed and maintained through a third-party vendor.

The scheduling process from cloud users submitting data to returning processing results can be represented as shown in Figure 3.

After the user submits the data to be executed to the cloud environment, the multidata is first processed, divided into sets of multiple subdata, and submitted to the data scheduling center. Then, according to the data scheduling algorithm, the data scheduling center establishes a mapping relationship between the divided subdatasets and the available resource sets of the resource management center to meet the resource requirements of each data execution so as to execute the data submitted by the user. During the execution of data, the dispatch center will update the resource status according to the execution of the data. It allocates idle resources to complete data execution to newly submitted or pending data. The execution result is fed back to the user until all subdata in the dataset submitted by the user are executed.

The biological immune system has a perfect recognition mechanism and pathogen protection function. It consists of multiple immune subsystems and completes the immune protection function through the interaction between the subsystems. The biological immune system can be divided into nonspecific immunity and specific immunity. Among them, nonspecific immunity is an innate protective function. It is a defense ability against pathogens produced by organisms gradually adapting to the external environment during evolution. Its resistance to pathogens is broad. When the biological system is invaded by external pathogens, it can quickly make resistance defenses. Specific immunity is a form of organism defense against a certain type of pathogens formed by the stimulation of antigenic substances through acquired infection or artificial inoculation defense. Specific immunity plays a powerful role in the immune function of biological systems. The biological immune system ensures its own safety through the coordination of various functions. The immune defense is the biological system's defense against external pathogens to prevent the organism from being infected. Immune stabilization renews senescent and damaged cells in an organism to maintain functional integrity. Immune surveillance realizes the monitoring of the state of cells in an organism to avoid abnormal cells. In the rapid development and application of biotechnology and artificial intelligence technology, the use of immune mechanism in the field of artificial intelligence has created a new research field, namely, artificial immune system. Artificial immunity can be used in scientific research and production applications to solve difficult or unsolvable problems in the current field. In recent years, in the research and application of machine learning, big data, and cloud computing, artificial immunity has shown its advantages and has been widely used.

RETRACTED

According to the above-mentioned related theories and immune principles of artificial immunity, the artificial immune algorithm is a biomimetic artificial intelligence algorithm summed up on the basis of biological immunity. The specific flow of the standard artificial immune algorithm is shown in Figure 4.

It can be seen from this process that the specific process of standard artificial immunization is as follows:

1. Identify the antigen; that is, transform the problem, and define an appropriate affinity function according to the relevant constraints of the problem.
2. To generate an initial antibody population, a certain number of initial antibody populations can be generated according to the scale of the problem to be solved.
3. Calculate the affinity between each antibody and antigen in the antibody population.
4. Determine whether the calculated antigen-antibody affinity satisfies the termination condition of the algorithm. If satisfied, the optimal solution can be obtained; otherwise, the algorithm continues to execute.
5. Calculate the concentration of effective antibody in the current population.
6. The antibody with higher affinity is cloned and mutated, and the clone size is inversely proportional to the antibody concentration to prevent local optimization.
7. Update the antibody population and go to (3) to continue executing the algorithm.

In the theoretical research and application in various fields, artificial immune algorithm is often used to solve some more complex problems. Two types of commonly used algorithms are described in the following.

### 3.1. Clone Selection Algorithm

The clone selection algorithm is an intelligent search algorithm formed according to this defense mechanism of cells in the organism. The algorithm simulates the process of defense matching between “nonself” antigenic substances and antibodies produced in the body and can find the optimal solution to the problem. The algorithm process is shown in Figure 5.

The specific process of the algorithm is roughly as follows:

1. Generating the initial antibody population for the algorithm: it can determine the initial size of the antibody to be generated according to the scale of the problem and randomly generate the corresponding number of antibodies.
2. Affinity calculation and antibody selection: according to the set affinity calculation function, the affinity of each antibody and antigen in the population is calculated. And according to the calculation results, high-affinity antibodies are screened to form excellent populations.
3. Clone operation: in order to find the optimal solution to the problem faster, clone the selected excellent population. The better the antibody clones, the more clones, and vice versa.
4. Mutation operation: in order to obtain better antibodies in the existing population, it is necessary to mutate the antibodies to obtain new antibodies. Because the better antibodies are close to the optimal solution, the antibodies with low affinity are subjected to a large number of mutations, and the relatively excellent antibodies are subjected to weaker mutations. After this operation, if better antibodies are produced in the population, the population is added to remove the same number of weaker antibodies.
5. Antibody memory: the excellent antibody is selected as the memory antibody in the new population, and it is regarded as the excellent solution in the second selection.
6. Determining whether the antibodies in the new population can meet the termination condition of the problem: if so, take the best antibody as the optimal solution to the problem; otherwise, update the antibody population, go to (2), and continue to execute the algorithm.

RETRACTED

### 3.2. Negative Selection Algorithm

The immune system can distinguish between “self” and “nonself” in the process of immunization to achieve the effect of eliminating “nonself” substances. Negative selection is to identify autologous cells and “nonself” cells by judging whether T cells react with self-proteins during the formation of T cells. If there is a reaction between them, it is a “nonself” substance and needs to be removed. The remaining cells are used by the immune system to defend against antigens. The negative selection algorithm is formed based on this discrimination mechanism, and its working principle is shown in Figure 6.

It can be known from the algorithm principle that, in the selection process, the candidate set is first matched and compared with the existing self-set. According to the matching result, the data that can match the self-set in the candidate set are discarded, and the data that cannot be matched are added to the detector set. The detection items are matched and compared with the obtained detector set, the detection items that can match the detector set are “nonself,” and the detection items that cannot match the detection items are self-identical. Therefore, the main process of the negative selection algorithm is as follows:

1. According to the problem to be solved, define the own string set S.
2. Randomly select the candidate set and compare it with the self-set S. The detector set *R* consists of candidate set elements that do not match S.
3. Compare the detection item with each detector in the detector set *R* in turn according to the comparison rule, and obtain the detection result.

## 4. Tourism Economic Data Scheduling Algorithm

Minimax optimization problem is as follows:

(1) $$\begin{array}{c} \min\;\Gamma \left(\zeta \right)=\min_{\mu =1}^{\omega }\text{Max }\delta_{\mu }\left(\zeta \right). \end{array}$$

Among them, *δ*_*μ*_(*ζ*) is a continuous differentiable function, and *ω* is a positive integer. However, the function Γ(*ζ*) is not differentiable, and the optimal solution to the problem cannot be obtained by using conventional mathematical optimization methods. Therefore, it is very difficult to solve this kind of problem numerically. The derivation of the maximum entropy function is as follows:

(2) $$\begin{array}{c} \Gamma \left(\zeta \right)=\overset{\omega }{\underset{\mu =1}{\max\;\delta_{\mu }\left(\zeta \right)}},\\ \Xi =\left\{\rho \in \Sigma^{\omega }:\rho_{\mu }\geq 0,\mu =1,2,\ldots ,\omega ,\sum_{\mu =1}^{\omega }\rho_{\mu }=1\right\}. \end{array}$$

So there is

(3) $$\begin{array}{c} \Gamma \left(\zeta \right)=\underset{\rho_{\mu }\in \Xi }{\max}\left(\sum_{\mu =1}^{\omega }\rho_{\mu }\delta_{\mu }\left(\zeta \right)\right),\\ \Gamma_{q}\left(\zeta \right)=\underset{\rho_{\mu }\in \Xi }{\max}\left(\sum_{\mu =1}^{\omega }\rho_{\mu }\delta_{\mu }\left(\zeta \right)-\frac{1}{q}\sum_{\mu =1}^{\omega }\rho_{\mu }\ln\;\rho_{\mu }\right),\\ \Gamma_{q}\left(\zeta \right)=\frac{1}{q}\ln\;\sum_{\mu =1}^{\omega }e^{q\delta_{\mu }\left(\zeta \right)}. \end{array}$$

And there are Γ(*ζ*) and Γ_*q*_(*ζ*) with the following properties:

(4) $$\begin{array}{c} 0\leq \Gamma_{q}\left(\zeta \right)-\Gamma \left(\zeta \right)\leq \frac{\ln\;\omega }{q}. \end{array}$$

According to this property, it can be seen from the definition of convergence that when *q*⟶*∞*, Γ_*q*_(*ζ*) uniformly converges to Γ(*ζ*). Therefore, when the value of *q* is relatively large, solving the optimization problem of Γ(*ζ*) can be transformed into the optimization problem of solving the differentiable function Γ_*q*_(*ζ*).

RETRACTED

Several common optimization methods are described as follows:

(1) Unconstrained optimization problem.
This type of problem can use mathematical methods to derive the function of the problem with respect to the variables. The optimal solution to the problem can be obtained by substituting the point where the derivative is 0 into the original function for comparison and verification.
(2) Optimization problem with equality constraints.
In this type of problem model, the solution for the objective function is constrained by equality conditions. The optimal solution for the objective function must satisfy the equality constraints to be a feasible solution. Assuming that the objective function of the problem is *δ*(*ζ*) and there are multiple constraint functions *χ*(*ζ*), the corresponding optimization problem with constraints can be expressed as follows:
  (5) $$\begin{array}{c} \left\{\begin{array}{c} \min.\\ \text{s.t.} \end{array}\right.\begin{array}{c} \delta \left(\zeta \right),\\ \chi_{\mu }\left(\zeta \right)=0,\;\left(\mu =1,2,\ldots ,\omega \right). \end{array} \end{array}$$
Among them, *χ*_*μ*_(*ζ*)=0,  (*μ*=1,2,…, *ω*) represents the *ω* equality constraints of the problem.
When solving the above problems, the commonly used method is the Lagrange multiplier method. Simply put, it is to multiply multiple equality constraints by the corresponding parameters, which together with the objective function of the problem form a Lagrangian function. By solving this _function, the optimal solution to the original problem can be obtained. For example, the Lagrangian function of problem (5) can be defined as follows:
  (6) $$\begin{array}{c} \varphi \left(\zeta ,\rho \right)=\delta \left(\zeta \right)+\sum_{\mu =1}^{\omega }\rho_{\mu }\chi_{\mu }\left(\zeta \right). \end{array}$$
Among them, *ρ*_*μ*_ is the constraint parameter of constraint *χ*_*μ*_(*ζ*).
When solving *φ*(*ζ*, *ρ*), the partial derivatives of the expressions can be obtained with respect to each variable, and the equations can be solved in parallel as follows:
  (7) $$\begin{array}{c} \left\{\begin{array}{c} \frac{\partial \varphi \left(\zeta ,\rho \right)}{\partial \zeta }=\frac{\partial \delta \left(\zeta \right)}{\partial \zeta }+\sum_{\mu =1}^{\omega }\rho_{\mu }\frac{\partial \chi_{\mu }\left(\zeta \right)}{\partial \zeta }=0,\\ \frac{\partial \varphi \left(\zeta ,\rho \right)}{\partial \rho_{1}}=\chi_{1}\left(\zeta \right)=0,\\ \begin{array}{c} •\\ •\\ • \end{array}\\ \frac{\partial \varphi \left(\zeta ,\rho \right)}{\partial \rho_{\omega }}=\chi_{\omega }\left(\zeta \right)=0. \end{array}\right. \end{array}$$
(3) KKT conditions for optimization problems with inequality constraints.

In the solution to optimization problems, there are often optimization problems with constraints of inequality conditions. Suppose that the objective function of the problem is *δ*(*ζ*), and the equality constraint function is *χ*(*ζ*) inequality. Then, the corresponding conditional constrained optimization problem can be expressed as follows:

(8) $$\begin{array}{c} \left\{\begin{array}{c} \min.\\ \text{s.t.} \end{array}\right.\begin{array}{c} \delta \left(\zeta \right),\\ \begin{array}{c} \chi_{\mu }\left(\zeta \right)=0,\;\left(\mu =1,2,\ldots ,\omega \right),\\ \varepsilon_{\nu }\left(\zeta \right)\leq 0,\;\left(\nu =1,2,\ldots ,\xi \right). \end{array} \end{array} \end{array}$$

Among them, *χ*_*μ*_(*ζ*)=0,  (*μ*=1,2,…, *ω*) represents the *ω* equality constraints of the problem, and *ε*_*ν*_(*ζ*) ≤ 0,  (*ν*=1,2,…, *ξ*) represents the *ξ* equality constraints of the problem.

RETRACTED

To find the optimal solution under such constraints, the Lagrangian function of problem (8) can be defined as follows:

(9) $$\begin{array}{c} \varphi \left(\zeta ,\rho ,\varpi \right)=\delta \left(\zeta \right)+\sum_{\mu =1}^{\omega }\rho_{\mu }\chi_{\mu }\left(\zeta \right)+\sum_{\nu =1}^{\xi }\varpi_{\mu }\varepsilon_{\mu }\left(\zeta \right). \end{array}$$

Among them, *ρ*_*μ*_ is the constraint parameter of constraint *χ*_*μ*_(*ζ*), and *ϖ*_*μ*_ is the constraint parameter of constraint *ε*_*μ*_(*ζ*).

When solving the optimal solution to this problem, the KKT (Karush–Kuhn–Tucker) optimization condition of this problem can be introduced. It is expressed as follows:

(10) $$\begin{array}{c} \left\{\begin{array}{c} \frac{\partial \varphi \left(\zeta a,\rho ,\varpi \right)}{\partial \rho }=0,\\ \rho_{\mu }\neq 0,\\ \varpi_{\nu }\geq 0,\\ \begin{array}{c} \varpi_{\nu }\varepsilon_{\nu }\left(\zeta \right)=0,\\ \chi_{\mu }\left(\zeta \right)=0,\\ \varepsilon_{\nu }\left(\zeta \right)\leq 0, \end{array} \end{array}\;\left(\mu =1,2,\ldots ,\omega ;\nu =1,2,\ldots ,\xi \right)\right.. \end{array}$$

The tourism economic data scheduling in the cloud environment is to establish a mapping from a tourism economic dataset Θ to a distributed resource set Π according to a certain scheduling strategy. It maps the tourism economic data nodes with dependencies to the heterogeneous resources in the cloud environment and denotes the mapping as Ξ : Θ⟶Π. When Ξ(Θ_*μ*_, Π_*ν*_)=0, it means that there is no mapping relationship between the data node Θ_*μ*_ and the resource node Π_*ν*_. When Ξ(Θ_*μ*_, Π_*ν*_)=1, it means that the data node Θ_*μ*_ is allocated to the resource Π_*ν*_.

In order to illustrate the scheduling model of the tourism economic data, the following description is made first.

First, for a data node Θ_*μ*_, the resource node Π_*ν*_ to be called must meet the following conditions before it can join the resource scheduling queue of the data node:

(11) $$\begin{array}{c} \left\{\begin{array}{c} \Theta_{\mu }\left(\gamma \left(\Sigma \right)\right)\leq \Pi_{\nu }\left(\Sigma \right),\\ \Theta_{\mu }\left(\gamma \left(\Lambda \right)\right)\leq \Pi_{\nu }\left(\Lambda \right),\\ \Theta_{\mu }\left(\gamma \left(Κ\right)\right)\leq \Pi_{\nu }\left(Κ\right). \end{array}\right. \end{array}$$

Among them, Σ represents the computing capability of resource node Π_*ν*_. Λ represents the storage capacity of resource node Π_*ν*_. Κ represents the network processing capability of the resource node Π_*ν*_. Θ_*μ*_(*γ*) represents the execution demand of data node Θ_*μ*_.

**Definition 1 .**

Assuming that data node Θ_*μ*_ is allocated to resource node Π_*ν*_, then according to the computational requirements, the computing time of data node Θ_*μ*_ on Π_*ν*_ is as follows:

(12) $$\begin{array}{c} \eta \left(\Theta_{\mu },\Pi_{\nu }\right)=\frac{\Theta_{\mu }\left(\gamma \right)}{\Pi_{\nu }\left(\Sigma \right)}. \end{array}$$

When a data node requests a resource node to execute data, only when all parent data of the data node completes execution and the resource node is idle and available, the data scheduler can allocate it so that the data node can obtain resources for execution. Therefore, the following definitions can be made.

**Definition 2 .**

The earliest time when a data node can obtain a resource node is

(13) $$\begin{array}{c} \kappa \left(\Theta_{\mu },\Pi_{\nu }\right)=\max\left\{\sigma \left(\Pi_{\nu }\right),\varsigma_{\max}\right\}. \end{array}$$

Among them, *σ*(Π_*ν*_) can obtain the earliest available time of resource node Π_*ν*_. When there is data to execute on the resource node, it can be considered that the time when the data is executed is obtained through this operation. *ς*_max_ is the maximum value of the total time to complete data execution and complete communication with the current data node in the data node's parent data node set. It can be calculated by the following calculation expression:

(14) $$\begin{array}{c} \varsigma_{\max}=\underset{\Theta_{q}\in \Theta_{\mu }\left(\tau \right)}{\max}\left\{\upsilon \left(\Theta_{q}\right)+\psi \left(\Theta_{\mu },\Theta_{q}\right)\right\}. \end{array}$$

Among them, *υ*(Θ_*q*_) can obtain the actual completion time of the parent data of the data node. Because the child data nodes in the tourism economic data must be executed after all the parent data nodes are executed, the actual completion time of the parent data node can be obtained when data node Θ_*μ*_ is executed. *ψ*(Θ_*μ*_, Θ_*q*_) is the communication time delay from the parent data node to the current data node.

RETRACTED

**Definition 3 .**

After the data node obtains the resource node, the resource cannot be released until the data is executed. Therefore, the earliest time for data to complete data execution on the resource node is as follows:

(15) $$\begin{array}{c} \theta \left(\Theta_{\mu },\Pi_{\nu }\right)=\kappa \left(\Theta_{\mu },\Pi_{\nu }\right)+\eta \left(\Theta_{\mu },\Pi_{\nu }\right). \end{array}$$

(a) Completion time constraints of tourism economic data nodes.
One measure of a data scheduling algorithm is how good it is in terms of data completion time. The final completion time of the data is an important aspect of the performance of the scheduling algorithm. For the data nodes in the tourism economic dataset, there are many resources in the cloud environment resource set that meet the scheduling requirements of the node. In order to obtain better scheduling performance, after the resource nodes are obtained according to the data nodes, the completion time for completing the execution of the data nodes can be used as a constraint condition. The completion time constraint function for matching between data nodes and resource nodes to complete data is defined as follows:
  (16) $$\begin{array}{c} \vartheta \left(\Theta_{\mu },\Pi_{\nu }\right)=\frac{\underset{\Pi_{ο}\in \Pi }{\max}\left\{\theta \left(\Theta_{\mu },\Pi_{ο}\right)\right\}-\theta \left(\Theta_{\mu },\Pi_{\nu }\right)+1}{\underset{\Pi_{ο}\in \Pi }{\max}\left\{\theta \left(\Theta_{\mu },\Pi_{ο}\right)\right\}-\underset{\Pi_{t}\in \Pi }{\min}\left\{\theta \left(\Theta_{\mu },\Pi_{t}\right)\right\}+1}. \end{array}$$
Among them, Π_*ο*_ and Π_*t*_ represent any resource nodes in the virtual resource pool.
(b) Cross-node transmission delay constraint.

In the process of data scheduling, due to the heterogeneity and distribution characteristics of resources in the cloud environment, the scheduling resources that meet the scheduling performance requirements are often located in different regions. When communicating or transmitting data between resource nodes in different regions, it is necessary to communicate through node routing. And the data nodes of tourism economic data have dependencies. When these data nodes need to schedule resource nodes in different regions, the overall performance of data scheduling will be affected due to the transmission delay of cross-node routing. Assume that the resource node where the data node is located is *α* and the resource node allocated by its parent data is *β* when the current data node is executed after the parent data of the data node is executed. The transmission delay constraint due to cross-nodes can be expressed by the following expression:

(17) $$\begin{array}{c} \beta \left(\Pi_{\mu },\Pi_{\nu }\right)=\frac{\underset{\Pi_{ο}\in \Pi }{\max}\left\{\alpha \left(\Pi_{ο},\Pi_{\nu }\right)\right\}-\alpha \left(\Pi_{\mu },\Pi_{\nu }\right)+1}{\underset{\Pi_{ο}\in \Pi }{\max}\left\{\alpha \left(\Pi_{ο},\Pi_{\nu }\right)\right\}-\underset{\Pi_{t}\in \Pi }{\min}\left\{\alpha \left(\Pi_{t},\Pi_{\nu }\right)\right\}+1}. \end{array}$$

Among them, *α*(Π_*μ*_, Π_*ν*_) is the communication transmission delay between resource node Π_*μ*_ and resource node Π_*ν*_.

RETRACTED

### 4.1. Antibody Gene Coding

The coding of antibody genes can represent the solution to the problem, and in the data scheduling problem, it can represent the matching scheme of data and resources. In the artificial immune algorithm of flow data, the array sequence corresponding to the data number and the resource number is used to represent the antibody gene code. The length of the antibody gene encoding array is equal to the total number of nodes in the stream data. Each array represents a scheduling strategy between data and resources. For example, an antibody gene encoding method between the flow data of 8 data nodes and 4 virtual resources can be expressed as shown in Tables 1 and 2.

The antibody gene coding arrays in Tables 1 and 2 are {3, 2, 4, 1, 4, 3, 1, 2}. The position of the character in the array represents the number of the data. The value of the corresponding character is the resource number for executing the corresponding data. For example, data node 1 executes on resource 3, data node 2 executes on resource 2, and data node 3 executes on resource 4. The corresponding resources are scheduled to execute the flow data according to the encoding in the string in turn.

RETRACTED

### 4.2. Antibody Population Initialization

In the cloud environment, for the scheduling problem of flow data of N data nodes and tourism economic data of *M* virtual resources, according to the coding method of antibody genes, the initial population of antibodies is a set of K integer arrays of length N. And the sequence of characters in each array is a number between 0 and M. According to the implementation characteristics of tourism economic data, and this paper considers the DAG structure of tourism economic data when initializing the antibody population. According to the structure of the data, the resource requirements of the upper nodes in the structure are given priority. The remaining nodes are then allocated resources in the resource sequence. In the tourism economic data, priority is given to randomly assigning resources to data node 1, data node 2, data node 3, and data node 4 in the first layer. Then, data node 5, data node 6, and data node 7 of the second layer allocate resources and randomly allocate resources according to the data level. Until K antibody array sets are generated, the initial antibody population of tourism economic data is formed.

### 4.3. Affinity Function

In the artificial immune algorithm, the selection of the affinity function plays an extremely important role in the process of screening out excellent antibodies and finally obtaining the optimal solution to the problem. In the process of antibody screening, affinity is used as an indicator of antibody screening throughout the entire algorithm process. Therefore, the determination of the affinity function will affect the performance of the entire artificial immune algorithm. In this paper, aiming at the heterogeneity of resources in the cloud environment and the characteristics between streaming data nodes in tourism economic data processing, when determining the affinity function in the algorithm, it comprehensively considers the influence of the completion time of tourism economic data nodes and the transmission delay across nodes on the selection of virtual resources for data. It introduces the comprehensive fitness function of data nodes to measure the fitness of any virtual machine resource performance to the current data. The comprehensive fitness function of data *μ* to virtual machine resource *ν* is expressed as follows:

(18) $$\begin{array}{c} Η\left(\Theta_{\mu },\Pi_{\nu }\right)=\vartheta \left(\Theta_{\mu },\Pi_{\nu }\right)*\Psi +\beta \left(\Theta_{\mu },\Pi_{\nu }\right)*\Delta . \end{array}$$

Among them,

(19) $$\begin{array}{c} \left\{\begin{array}{c} \Psi =\frac{|\Theta_{o}\left(\tau \right)|*\sum_{ο=1}^{\omega }\eta \left(\Theta_{o},\Pi_{\nu }\right)}{|\Theta_{o}\left(\tau \right)|*\left(\sum_{ο=1}^{\omega }\eta \left(\Theta_{o},\Pi_{\nu }\right)\right)+\omega \sum_{\Theta_{t}\in \Theta_{o}\left(\tau \right)}\psi \left(\Theta_{\mu },\Theta_{t}\right)},\\ \Delta =\frac{\omega \sum_{\Theta_{t}\in \Theta_{o}\left(\tau \right)}\psi \left(\Theta_{\mu },\Theta_{t}\right)}{|\Theta_{o}\left(\tau \right)|*\left(\sum_{ο=1}^{\omega }\eta \left(\Theta_{o},\Pi_{\nu }\right)\right)+\omega \sum_{\Theta_{t}\in \Theta_{o}\left(\tau \right)}\psi \left(\Theta_{\mu },\Theta_{t}\right)}. \end{array}\right. \end{array}$$

RETRACTED

### 4.4. Cloning Operation

According to the affinity function defined in (3), each antibody in the antibody population can be calculated, that is, the affinity of the scheduling scheme for the problem. According to the calculation results, the antibody with a higher affinity is selected for cloning operation, and the size of the clone is proportional to the affinity of the antigen-antibody. A high affinity indicates that it is closer to the optimal solution to the problem, and the proportion of such excellent solutions should be increased. Therefore, cloning operations can be used to increase the proportion of relatively excellent antibodies in the antibody population, thereby expanding the concentration of excellent antibodies.

### 4.5. Gene Recombination

In the experiment, the tourism economic data scheduling algorithm based on artificial immune algorithm (referred to as AITSA) in this paper is compared with the genetic algorithm (GA) under the same experimental conditions for the scheduling of tourism economic data to verify the effectiveness of this algorithm. For the accuracy of the experimental results, 20 experiments were performed in each type of comparison, and the average value was used as the comparison value. The relevant parameter settings of the algorithm during the experiment are shown in Tables 3 and 4.

The purpose of the tourism economic data scheduling algorithm is to reasonably schedule the tourism economic data nodes to the resource nodes for execution, improve the execution efficiency of the entire tourism economic data, and shorten the data completion time. In the experiment process, mainly in the same operating environment, the tourism economic scheduling model based on artificial immune algorithm and the genetic algorithm (GA) were compared in terms of data completion time and algorithm execution speedup ratio, and then the performance differences of the two algorithms were compared. In order to avoid the influence of multiple data and different queuing rules on the algorithm comparison, in the process of this experiment, one piece of tourism economic data is submitted each time, and the performance of the two algorithms under different node scales is compared.

RETRACTED

In order to compare the algorithm execution performance of the AITSA algorithm and the GA algorithm under different data node scales, during the experiment, the node scales of the tourism economic data were set to 10, 20, 40, 60, 80, and 100 in turn. In the experiment, in order to highlight the difference in the execution effect of the two algorithms, the demand parameter of the data node is set to a value with a large difference. The data completion time of the two algorithms is shown in Figure 7.

Figure 7 shows that as the number of data nodes increases, the overall completion time of tourism economic data generally tends to rise. During the experiment, in order to ensure the accuracy of the results, the method of obtaining the average value of multiple experiments was adopted. The parameters of multiple experiments under the same experimental conditions do not change, and the experimental results are not biased when the scale of data nodes is small. When the scale of data nodes is large, there will be a small amount of deviation due to the limitations of experimental hardware conditions. However, in the experimental results with large data nodes, the completion time value is also large, and a small deviation change will not affect the experimental results.

The GA algorithm and AITSA algorithm are used to conduct tourism economic data scheduling experiments under different data node scales. The acceleration ratio of the experimental results is shown in Figure 8.

It can be seen from Figure 8 that when the scale of data nodes is small, the acceleration ratio of the AITSA algorithm is slightly higher than that of the GA algorithm, but the difference is not obvious. With the increase in node size, the difference between the speedup ratios of the two algorithms shows an increasing trend. It shows that, with the increase of scale, the difference in speedup ratio between the two algorithms keeps increasing. Under different data node scales, the acceleration of the AITSA algorithm has certain advantages compared with the GA algorithm. It can be seen that the tourism economic data scheduling algorithm based on artificial immune calculation in this paper has higher execution efficiency.

In the experiment process, in order to facilitate the comparison and representation, the average sharding data scheduling algorithm is denoted as ESDSA, and the data sharding-based data scheduling strategy proposed in this paper is denoted as SDSA. Because of the scheduling strategy generated by the SASA algorithm proposed in this paper, the number of resource nodes that are requisitioned varies with the performance of resource nodes and the minimum slicing granularity of data-related data. For the fairness of the algorithm comparison, the data volume, data slicing granularity, and the number of available resources each time are set to the same fixed values during the experiment. For the accuracy of the experimental results, 20 experiments were performed in each type of comparison, and the average of the 20 experimental results was taken as the comparison value. The relevant parameter settings in the algorithm are shown in Table 5.

RETRACTED

The following is a comparison of the data response time of the two algorithms under the conditions of different resource node scales and different data volumes as performance indicators.

In order to compare the performance of the SDSA algorithm and ESDSA algorithm in resource node environments of different scales, during the calling process of the algorithm, the scale of resource nodes is set to 10, 20, 50, 100, 150, and 200 in turn. In the experiment, in order to reflect the difference between the two algorithms, the performance parameters of the resource nodes are set to values with large differences. Through experiments, the response time of data using the two algorithms under different resource node scales is shown in Figure 9.

It can be seen from Figure 9 that when the scale of resource nodes is less than 100, the data completion time of the data fragmentation data scheduling algorithm (ESDSA) proposed in this paper is shorter than that of the data average fragmentation data scheduling algorithm. When the resource scale is greater than 100, the data completion times of the two algorithms are similar. This is because ESDSA can fully utilize the processing performance of resources when available resources are limited. The amount of data shards is divided proportionally according to the performance of the resource nodes so that the processing completion time of each shard is relatively close so that the overall data completion time is faster. When the scale of available resources is large, the number of data fragments increases accordingly, the amount of fragmented data allocated to each resource node is relatively small, and the data are completed faster. The two algorithms are not very different. It can be seen that, in data scheduling with a limited scale of available resources, the SDSA algorithm outperforms the ESDSA algorithm.

In order to compare the performance of the two algorithms at different times, the resource scale is set to a fixed value in the experiment, and the amount of submitted data is set to 1000, 2500, 5000, 10000, 15000, and 20000 in turn. For data with different amounts of data, the response times of the two algorithms are shown in Figure 10.

RETRACTED

It can be seen from Figure 10 that when the amount of data is small, the amount of data sharded to the resource nodes is also small due to the small amount of processing. There is not much difference in the completion time of the two algorithms. However, when the data scale is large, SDSA can make good use of resource nodes with better performance. It shows a great advantage in terms of completion time.

## 5. Discussion

The rise of cloud computing has changed the way traditional IT services are provided, people's understanding of how resources are used, and the way the Internet operates and makes money. Cloud computing provides a convenient service method for people to use services anytime and anywhere through the Internet. The service provided by the cloud computing system to the user is based on the resource call in the cloud environment. The job submitted by the user is submitted to the cloud environment, and the data is processed and fed back by the resources in the cloud environment. Due to the large scale, heterogeneous sharing, and dynamic changes of cloud resources, data scheduling in the cloud environment is an extremely complex process. Data scheduling in the same scenario often requires a corresponding scheduling strategy to better complete data execution. In addition, the use of cloud computing technology brings certain limitations to the selection of this research. The fitness function in different scheduling scenarios will vary according to the actual scenario. The fitness function in the workflow task scheduling algorithm in this paper is not necessarily suitable for other application scenarios.

## 6. Conclusion

In the scheduling scenario of tourism economic data, the cross-regional distribution of resources will affect the communication transmission efficiency between data nodes and the final completion time of data. Data processing data scheduling problem requires a reasonable data fragmentation strategy and resource scheduling strategy to improve the efficiency of data processing. Based on these two application scenarios, this paper studies the tourism economic data scheduling algorithm and the data sharding data scheduling algorithm to improve the data execution efficiency in the cloud environment. In the scheduling scenario of data processing data, the existing sharding methods cannot well solve the problems of data sharding and resource requisition in the cloud environment. For practical application scenarios, in order to make full use of the computing performance and network performance of available resources, this paper proposes a data scheduling strategy based on data sharding. According to the performance of resource nodes and the segmentation granularity of the data to be processed, an ideal segmentation strategy can be obtained. The data to be processed is then sharded twice according to the sharding strategy to obtain the final sharding strategy. The experimental verification shows that this strategy can significantly improve the data execution efficiency. In addition, the use of cloud computing technology brings certain limitations to the selection of this research. The fitness function in different scheduling scenarios will vary according to the actual scenario. The fitness function in the workflow task scheduling algorithm in this paper is not necessarily suitable for other application scenarios.

RETRACTED

## Figures and Tables

**Figure 1:** Architecture of cloud computing.

**Figure 2:** Types of cloud computing services.

**Figure 3:** Data scheduling process in cloud environment.

**Figure 4:** Flowchart of artificial immunization.

**Figure 5:** Clone selection algorithm flow.

**Figure 6:** Principle of negative selection algorithm.

**Figure 7:** Comparison of data completion time of two algorithms under different data node scales.

**Figure 8:** Comparison of the speedup ratio of the two algorithms under different data node scales.

**Figure 9:** Response time of different algorithms under different resource node scales.

**Figure 10:** Response time of the two algorithms under different amounts of data.

**Table 1:** Examples of antibody gene coding methods.

Data encoding	1	2
Resource encoding	3	2
Data encoding	3	4
Resource encoding	4	1

**Table 2:** Examples of antibody gene coding methods.

Data encoding	5	6
Resource encoding	4	3
Data encoding	7	8
Resource encoding	1	2

**Table 3:** Experiment-related parameter settings.

	Parameter	Value/range
1	Number of resource nodes	30
2	Data node size	10–100
3	Data length	10000–50000

**Table 4:** Experiment-related parameter settings.

	Parameter	Value/range
4	Resource node region span	0–5
5	Resource node computing capability	200–1000
6	Resource bandwidth	20–100

**Table 5:** Algorithm-related parameter settings.

	Parameter	Value/range
1	Number of resource nodes	200
2	The amount of data	1000–20000
3	Minimum segmentable granularity of data	10–100
4	Amount of data	1–200
5	Data bandwidth requirements	10–100

## Data Availability

No datasets were generated or analyzed during this study.

## References

[1] Chen X., Wang L. (2017). Exploring fog computing-based adaptive vehicular data scheduling policies through a compositional formal method-PEPA. *IEEE Communications Letters*.

RETRACTED

[2] Verma L. P., Kumar M. (2017). An adaptive data chunk scheduling for concurrent multipath transfer. *Computer Standards & Interfaces*.

[3] Dang S., Tang W. (2021). Real-time data scheduling of flexible job in papermaking workshop based on deep learning and improved fuzzy algorithm. *Mobile Information Systems*.

[4] Luo W., Gu B., Lin G. (2018). Communication scheduling in data gathering networks of heterogeneous sensors with data compression: algorithms and empirical experiments. *European Journal of Operational Research*.

[5] Joo C., Kang S. (2017). Joint scheduling of data transmission and wireless power transfer in multi-channel device-to-device networks. *Journal of Communications and Networks*.

[6] Zhang Y., Cui L., Zhang Y. (2017). A stable matching based elephant flow scheduling algorithm in data center networks. *Computer Networks*.

[7] Huang J., Xu L., Duan Q., Xing C., Luo J., Yu S. (2017). Modeling and performance analysis for multimedia data flows scheduling in software defined networks. *Journal of Network and Computer Applications*.

[8] Durazo-Cardenas I., Starr A., Turner C. J. (2018). An autonomous system for maintenance scheduling data-rich complex infrastructure: fusing the railways’ condition, planning and cost. *Transportation Research Part C: Emerging Technologies*.

[9] Xu G., Bai Y., Pan Q., Huang Q., Yang Y. (2017). Data verification tasks scheduling based on dynamic resource allocation in mobile big data storage. *Computer Networks*.

[10] Kostenko V. A., Plakunov A. V. (2017). Ant algorithms for scheduling computations in data centers. *Moscow University Computational Mathematics and Cybernetics*.

[11] Sharma V. K., Verma L. P., Kumar M. (2019). CL-ADSP: cross-layer adaptive data scheduling policy in mobile ad-hoc networks. *Future Generation Computer Systems*.

[12] Zhou D., Sheng M., Luo J., Liu R., Li J., Han Z. (2019). Collaborative data scheduling with joint forward and backward induction in small satellite networks. *IEEE Transactions on Communications*.

[13] Rawat M. A., Singh H. H., Syed A. (2018). A Survey on data scheduling and its analysis on big data. *SSRN Electronic Journal*.

[14] Zhang G. (2017). Simulation research on the cloud computing data scheduling and distribution technology based on balanced energy consumption modelling. *Boletin Tecnico/Technical Bulletin*.

[15] Kaushal P., Sinha S., Sinha V. K. (2021). Virtual machine placement in cloud computing: challenges, research gaps, and future. *International Journal of Wireless and Ad Hoc Communication*.

RETRACTED

[16] Ibrahim E., Salwa H. M., Moustafa A. (2020). A lightweight privacy preserving keyword search over encrypted data in cloud computing. *Journal of Cybersecurity and Information Management*.

[17] Lu P., Zhu Z. (2017). Data-oriented task scheduling in fixed- and flexible-grid multilayer inter-DC optical networks: a comparison study. *Journal of Lightwave Technology*.

[18] Qi Y., Cheng P., Chen J. (2017). Optimal sensor data scheduling for remote estimation over a time-varying channel. *IEEE Transactions on Automatic Control*.

[19] Chen H., Zhai B., Wu J., Du C., Li J. (2020). A satellite observation data transmission scheduling algorithm oriented to data topics. *International Journal of Aerospace Engineering*.

[20] Cohen R., Polevoy G. (2019). Inter-datacenter scheduling of large data flows. *IEEE Transactions on Cloud Computing*.

[21] Che H., Bai Z., Zuo R., Li H. (2020). A deep reinforcement learning approach to the optimization of data center task scheduling. *Complexity*.

[22] Gao Y., Li X., Li J., Gao Y. (2019). Distributed and efficient minimum-latency data aggregation scheduling for multichannel wireless sensor networks. *IEEE Internet of Things Journal*.

[23] Comsa I. S., Zhang S., Aydin M. E. (2018). Towards 5G: a reinforcement learning-based scheduling solution for data traffic management. *IEEE Transactions on Network and Service Management*.

[24] Convolbo M. W., Chou J., Hsu C. H., Chung Y. C. (2018). GEODIS: towards the optimization of data locality-aware job scheduling in geo-distributed data centers. *Computing*.

[25] Nguyen N. T., Liu B. H., Pham V. T., Liou T. Y. (2018). An efficient minimum-latency collision-free scheduling algorithm for data aggregation in wireless sensor networks. *IEEE Systems Journal*.

[26] admin A., KiruthikaS K., Nithya S., Poornima B., Dharanya S. D., Kiruthika S. K. (2022). Enhancement of cloud user data access security entrusted to AI face recognition techniques. *Journal of Cognitive Human-Computer Interaction*.

[27] Hong H., Zhao W., Liu R., Kadoch M. (2020). Space-air-ground IoT network and related key technologies. *IEEE Wireless Communications*.

[28] Lv Z., Song H. (2020). Mobile Internet of things under data physical fusion technology. *IEEE Internet of Things Journal*.

